RETRACTED

# Stromal vascular fraction cells for the treatment of critical limb ischemia: a pilot study

**DOI:** 10.1186/s12967-017-1243-3

**Published:** 2017-06-19

**Authors:** Adas Darinskas, Mindaugas Paskevicius, Gintaras Apanavicius, Gintaris Vilkevicius, Liutauras Labanauskas, Thomas E. Ichim, Rytis Rimdeika

**Affiliations:** 1 Laboratory of Immunology, National Cancer Institute, Santariskiu Str. 1, 08660 Vilnius, Lithuania; 2 Department of Vascular Surgery, Vilnius City Clinical Hospital, Antakalnio Str. 57, 10207 Vilnius, Lithuania; 3 Northway Medical and Surgical Center, S.Zukausko Str. 19, 08234 Vilnius, Lithuania; 4 Clinics of Cardiovascular Diseases, Vilnius University, Santariskiu Str. 2, 08661 Vilnius, Lithuania; 5 Department of Plastic and Reconstructive Surgery, Lithuanian University of Health Sciences, Medical Academy, University Clinics of Kaunas, Eiveniu Str. 2, 50009 Kaunas, Lithuania; 6 Immune Advisors LLC, San Diego, CA 92121 USA

**Keywords:** Angiogenesis, Arteriosclerosis obliterans, Stromal vascular fraction cells, Critical limb ischemia

## Abstract

**Background:**

Cell-based therapy is being explored as an alternative treatment option for critical limb ischemia (CLI), a disease associated with high amputation and mortality rates and poor quality of life. However, therapeutic potential of uncultured adipose-derived stromal vascular fraction (SVF) cells has not been evaluated as a possible treatment. In this pilot study, we investigated the efficacy of multiple injections of autologous uncultured adipose-derived SVF cells to treat patients with CLI.

**Methods:**

This study included 15 patients, from 35 to 77 years old, with rest pain and ulceration. SVF cells were injected once or twice in the ischemic limb along the arteries. Digital subtraction angiography was performed before and after cell therapy. The clinical follow up was carried out for the subsequent 12 months after the beginning of the treatment.

**Results:**

Multiple intramuscular SVF cell injections caused no complications during the follow-up period. Clinical improvement occurred in 86.7% of patients. Two patients required major amputation, and the amputation sites healed completely. The rest of patients achieved a complete ulcer healing, pain relief, improved ankle-brachial pressure index and claudication walking distance, and had ameliorated their quality of life. Digital subtraction angiography performed before and after SVF cell therapy showed formation of numerous vascular collateral networks across affected arteries.

**Conclusion:**

Results of this pilot study demonstrate that the multiple intramuscular SVF cell injections stimulate regeneration of injured tissue and are effective alternative to achieve therapeutic angiogenesis in CLI patients who are not eligible for conventional treatment.

RETRACTED

Trial registration number at ISRCTN registry, ISRCTN13001382. Retrospectively registered at 26/04/2017.

## Background

Peripheral arterial disease (PAD) is a major health care problem in our aging society. It results in obstruction of the blood supply to the lower or upper extremities. Intermittent claudication and rest pain are the main symptoms of limb ischemia. Critical limb ischemia (CLI) is the most advanced stage of PAD. It often coincides with ischemic ulceration and/or gangrene [1], and significantly decreases a patient’s quality of life. It is difficult to manage using current treatment modalities. Although several therapies, including medical and surgical procedures, may reduce patients’ symptoms and improve the condition of their limbs, a lot of patients are not candidates for surgery or percutaneous transluminal angioplasty (PTA). 25% of CLI patients requires a major amputation of a limb within 1 year after diagnosis [2]. It has been recently shown that cell-based therapies using bone marrow mononuclear cells (BM-MNCs), peripheral blood mononuclear cells (PB-MNCs) and bone marrow-derived mesenchymal stem cells (BM-MSCs) have effective outcomes in patients with CLI [1–5]. Nevertheless, the availability of an easily accessible cell source may greatly facilitate the development of new cell-based therapies. Cells residing in stroma of adipose tissue are now recognized as an accessible, abundant, and reliable source of various adult stem cells suitable for tissue engineering and regenerative medicine applications [6]. Adipose tissue is one of the most accessible tissues by mild operation and the only tissue in the human body that can be removed without leaving a functional defect. A vast amount of the stromal vascular fraction (SVF) in adipose and connective tissues can be easily obtained from patients using conventional liposuction and isolation methods [7]. The SVF consists of a heterogeneous mesenchymal population of cells that includes not only adipose stromal, hematopoietic stem and progenitor cells but also endothelial cells, erythrocytes, fibroblasts, lymphocytes, monocyte/macrophages and pericytes [8, 9]. During the past decade, the number of scientific publications related to preclinical and clinical use of adipose-derived stromal/stem cells (ASCs) has increased dramatically. A group of scientists in a clinical survey with SVF cells and more than 1000 patients treated, have shown that adipose tissue without substantial manipulation is beneficial even in orthopedic field [10]. A pilot study conducted by Lee et al. showed that ASC implantation could be a safe alternative to achieve therapeutic angiogenesis in CLI patients [11]. However, the therapeutic potential of uncultured SVF cells for CLI patients has not been investigated.

RETRACTED

The muscle tissue where the therapeutic cells are injected is, in fact, connective tissue, like the SVF cells themselves. That classifies this therapy as homologous, which, in the light of regulatory concerns about application of SVF cells in the European Union, is an important fact to point out.

In this study we aimed to evaluate the therapeutic potential of autologous, uncultured, readily available and easily isolated adipose-derived SVF cells injected directly into ischemic limb of patients with CLI who are not eligible for conventional treatment modalities.

## Methods

### Patients

Fifteen patients (from 35 to 77 years old) with CLI were enrolled in this study, which was conducted between April 2014 and May 2015. All patients were suffering from arteriosclerosis obliterans (ASO). Surgical bypass and/or PTA were not possible for all patients. Surgical amputation was the only treatment option for these patients who were suffering from rest pain (all cases) and ulcers (cases 1, 7, 8, 11, 12, 15), and pregangrene of two fingers (case 6). One patient (case 11) had already undergone minor amputation in the limb. Characteristics of the patients are shown in Table 1. All patients provided written informed consent and, after approval by the medical ethics committee of Vilnius City Clinical Hospital and the rule of compassionate use, underwent the SVF cell therapy. All patients had undergone angiography before and after SVF cell therapy. The clinical efficacy was evaluated by assessing arterial revascularization, pain relief, ulcer healing, walking distance and changes in ankle-brachial pressure index (ABI).

**Table 1:** Patients’ characteristics

Case	Age/gender	Diagnosis	Ulcer	Claudication (m)	Risk factors
1 (L)	35/M	ASO	+, non-healing	100–150	–
2 (R)	70/M	ASO	−	100–150	Smoking
3 (L)	68/M	ASO	−	100–150	Smoking
4 (L)	52/M	ASO	−	150–200	DM
5 (R)	59/M	ASO	−	50–100	DM, smoking
6 (Lu)	77/F	ASO	Pregangrene of two fingers	–	–
7 (L)	77/F	ASO	+, non-healing	100–150	DM
8 (R)	67/M	ASO	+	50–100	DM, smoking
9 (L)	60/F	ASO	−	100–150	DM, obesity
10 (R)	68/F	ASO	−	150–200	DM, obesity
11 (L)	60/M	ASO	+, non-healing	50–100	DM, obesity
12 (R)	56/M	ASO	+	150–200	DM, smoking
13 (L)	67/M	ASO	−	200–250	–
14 (R)	72/F	ASO	−	150–200	–
15 (R)	64/M	ASO	+	50–100	DM, smoking

*Lu* left upper limb, *L* left lower limb, *R* right lower limb, *ASO* arteriosclerosis obliterans, *DM* diabetes mellitus

### Adipose tissue collection

Adipose tissue was collected using 3 mm inner diameter cannula with three pyramidal order holes in the end. Cannula was used with 50 ml luer lock syringe (BD) and vacuum was made with the help of surgeon’s finger aspiration force. All adipose tissue was collected from abdomen area, under local anesthesia with lidocaine and adrenaline. Minimum amount of collected tissue was 40 ml.

RETRACTED

### SVF cell isolation

The lipoaspirate was washed within 12 h of collection with plenty of physiological solution and gentamicin (80 mg/l). Adipose fraction was cut using specially produced blend mesh to avoid usage of collagenase. A mechanical stainless steel two-bladed mill placed in a cylinder 5 cm in diameter and equipped with a metal 3 mm diameter mesh was used to mechanically disrupt the adipose tissue. The mill was rotated at speed not exceeding 260 rpm. Each fraction was minced three times and remaining homogenous lipoaspirate was centrifuged for 7 min at 850*g* in 50 ml falcon tubes. The upper fraction containing adipocytes was discarded, and the pellet was washed once with physiological solution and prepared for injections. Cell densities were determined by counting in a Neubauer’s hemocytometer, and cell viability was assessed using Trypan blue exclusion assay.

### Injection of SVF cells

Cells were prepared in 20 ml luer lock syringes (BD). Cells were diluted in physiological solution and autologous serum of the patient. Minimum amount of viable cells per one syringe applied was 20 million. Application consisted of at least 30 injections per one 20 ml syringe. Secondary injections were performed 2 months after first application of cells.

## Results

Multiple intramuscular SVF cell injections did not cause any complications in any of the patients during 5 days of hospitalization and all follow-up period. Overall, 86.7% of patients showed clinical improvement. Two patients (cases 10, 15) underwent a major amputation, 1 and 2 weeks after SVF cell therapy. The rest of patients reported either diminished or decreased rest pain at 12 weeks after SVF cell treatment. Table 2 shows the outcomes of SVF cell therapy. Ulceration was completely cured or improved in limbs of all patients suffering from ulcers after SVF cell therapy (Figs. 1, 3). No ulcer recurrence was observed in any of the patients during the follow-up period. 86.7% of patients showed improvement in walking distances. The ankle-brachial index (ABI) was improved from 17 to 48% at 12 months after SVF cell therapy, and the ABI was still higher 2 years later for all the patients. Digital subtraction angiography (DSA) performed before and after SVF cell therapy showed formation of numerous vascular collateral networks across affected arteries (Figs. 1, 2). None of the patients died during the follow-up period. The survival rate and freedom from major amputation of the limb at 24 months after SVF cell therapy were 100 and 86.7%, respectively.

RETRACTED

**Table 2:** SVF cell therapy and outcomes

Case	Age/gender	Diagnosis	Cells (mln.) administered per procedure (numbers of procedure)	Time after procedure (months)	Clinical symptom, ulcer healing	Claudication (m)	ABI improvement (%)
1 (L)	35/M	ASO	40 (2)	12	Improved, ulcer healed	500–600	48
2 (R)	70/M	ASO	56 (2)	12	Improved	300–350	23
3 (L)	68/M	ASO	32 (1)	12	Improved	250–300	18
4 (L)	52/M	ASO	55 (2)	12	Improved	400–450	40
5 (R)	59/M	ASO	38 (2)	12	Improved	300–350	35
6 (Lu)	77/F	ASO	45 (2)	12	Improved	–	–
7 (L)	77/F	ASO	42 (1)	12	Improved, ulcer healed	150–200	17
8 (R)	67/M	ASO	56 (2)	12	Improved, ulcer healed	200–250	29
9 (L)	60/F	ASO	36 (2)	12	Improved	300–350	37
10 (R)	68/F	ASO	32 (1)	1 week	Major amputation, wound healed	–	–
11 (L)	60/M	ASO	43 (2)	12	Improved, ulcer healed	300–350	25
12 (R)	56/M	ASO	51 (1)	12	Improved, ulcer healed	300–350	23
13 (L)	67/M	ASO	39 (2)	12	Improved	300–350	28
14 (R)	72/F	ASO	33 (1)	12	Improved	250–300	25
15 (R)	64/M	ASO	34 (1)	2 weeks	Major amputation, wound healed	–	–

*Lu* left upper limb, *L* left lower limb, *R* right lower limb, *ASO* arteriosclerosis obliterans

**Fig. 1:** Collateral vessel formation and ulcer healing after SVF cell therapy. Case 1: digital subtraction angiography (DSA) images before (**A**, **C**) and after SVF cell injections (**B**, **D**). Collateral vessel formation was increased in the knee, upper tibia, and lower tibia at 7 months after SVF cell therapy (**B**, **D**). Ulcer before treatment (**E**) and completely healed ulcer at 5 months after SVF cell injections (**F**)

**Fig. 2:** Collateral vessel formation after SVF cell therapy. Case 6: DSA images before (**A**) and 10 months after SVF cell injections (**B**). Images of occluded limb right after SVF administration (**C**) and 10 months after SVF cell injections (**D**)

**Fig. 3:** Wound healing after SVF cell therapy. Case 11: non-healing ulcer before treatment (**A**) and completely healed ulcer at 2 months after SVF cell injections (**B**). Case 7: non-healing ulcer before treatment (**C**) and improved healing ulcer at 5 months after SVF cell injections (**D**)

## Discussion

In the last decade cell-based therapies have been investigated as a promising treatment option for patients with CLI who are refractory to other treatment modalities. It provides encouraging therapeutic possibilities to enhance the repair of damaged or diseased tissues in CLI patients. Several studies have suggested beneficial effects of autologous BM-MSC based therapies [12, 13]. However, the percentage of MSCs in bone marrow is quite low and decreases with age [14]. Furthermore, after isolation, BM-MSCs need 2–3 weeks of in vitro culture to reach an amount sufficient for transplantation. Moreover, bone marrow suction is an invasive procedure. These drawbacks limit the possibility of wide clinical application of BM-MSCs [15]. In addition, the neovascularization capacity of transplanted BM-MNCs is reduced with aging; therefore this cell treatment is less appropriate in the older patients [16]. Last but not least, meta-analysis of randomized placebo controlled trials showed no advantage of bone marrow derived cell therapy on the primary outcome measures of amputation, survival, and amputation free survival in CLI patients [17]. Compared with bone marrow, subcutaneous adipose tissue can provide enough dosage for therapy without cell culture. This tissue is now recognized as an abundant and accessible source of multipotent stromal cells suitable for regenerative medicine [18]. Nevertheless, adipose tissue is routinely discarded as a medical waste. In this pilot study, we used autologous uncultured adipose-derived SVF cells as a potential treatment option for patients with CLI. Obtained results show the beneficial role of SVF cell therapy in reducing the rate of major amputations and improving quality of life in CLI patients. 86.7% of treated patients avoided the amputation of limbs. Previously it was demonstrated that SVF cell therapy accelerated diabetic wound healing [19]. In our study, complete wound healing occurred in all SVF cell—treated CLI patients. Previous studies have shown that ASCs exert their effects mainly via paracrine mechanisms and make beneficial contributions to tissue repair, regeneration and immunomodulation [11, 20, 21]. We have shown that injection of SVF cells is an effective way to promote healing of ulcer and skin regeneration. Moreover, this study, for the first time, showed that injections of uncultured SVF cells could accelerate angiogenesis. Digital subtraction angiography performed before and after SVF treatment showed that the transformation of preexistent collateral arterioles into functional collateral arteries occurred in CLI patients. The principle that justifies the therapeutic application of stem cells is the restoration of vascular cellularity, the control and the support of the newly formed vessels, which ensure an adequate supply of oxygen in critical ischemic areas [22]. Previous researchers have reported that SVF cells could secrete various angiogenic growth factors in vitro and enhance neovascularization of ischemic tissue in vivo [23, 24]. Our data supports previously published reports showing that SVF cells promote angiogenesis and tissue repair. In a study performed by Sheng et al., enhanced angiogenesis and cell proliferation were observed in the tissue treated by transplantation of SVF [15]. We used uncultured SVF cells directly injecting them into ischemic limb. Injections were placed along the occluded native arteries, because the density of preformed collaterals is highest in parallel orientation to the axial arteries. This is the preferred location for collateral growth [22]. Moreover, we suppose that uncultured heterogeneous SVF cells can be more effective than a purified cell population due to the fact that heterogeneous population contains fibroblasts, stem cells, endothelial cells, pericytes, mast cells, preadipocytes, smooth muscle cells, macrophages, and progenitor cells, which are known to accelerate wound healing [15]. SVF cells injected near the wound could not only stimulate host cells around the wound, but also provide growth factors and extracellular matrix. The principle of intramuscular injection is the creation of a cell depot with paracrine activity in the ischemic area [22]. Moreover, in order to obtain more beneficial effect, we diluted SVF cells with autologous serum, which also contains growth factors and cytokines. The results obtained from this pilot study have demonstrated the beneficial role of SVF cell therapy in reducing the rate of amputations, reducing pain, improving ABI and overall quality of life in CLI patients.

RETRACTED

## Conclusion

Our data indicate that uncultured SVF cells diluted with autologous serum represent a potent therapeutic combination for CLI patients. The multiple intramuscular SVF cell injections are effective alternative to achieve therapeutic angiogenesis in CLI patients for which surgical bypass and/or PTA are not possible, and that this treatment modality is appropriate and safe. Bearing in mind the easy procedure of cell isolation and preparation, SVF cells may provide a promising therapeutic option for CLI. However, to establish this cell therapy as a standard treatment, more investigation with a larger number of patients is necessary.

## Abbreviations

ABI: ankle-brachial pressure index
ASCs: adipose-derived stromal/stem cells
ASO: arteriosclerosis obliterans
BM-MNCs: bone marrow-derived mononuclear cells
BM-MSCs: bone marrow-derived mesenchymal stem cells
CLI: critical limb ischemia
DSA: digital subtraction angiography
MSCs: mesenchymal stem cells
PAD: peripheral artery disease
PB-MNCs: peripheral blood mononuclear cells
PTA: percutaneous transluminal angioplasty
SVF: stromal vascular fraction
